# Downregulation of miR-3934 in Peripheral Blood Mononuclear Cells of Asthmatic Patients and Its Potential Diagnostic Value

**DOI:** 10.1155/2021/8888280

**Published:** 2021-01-09

**Authors:** Wenyu Wang, Jing Wang, Hong Chen, Xiaofei Zhang, Kaiyu Han

**Affiliations:** ^1^Department of Respiratory and Critical Medicine, The Second Affiliated Hospital of Harbin Medical University, China; ^2^Department of Respiratory Medicine, Harbin Chest Hospital, China

## Abstract

**Background:**

The present study focused on the potential clinical significance of miR-3934 in the occurrence and development of asthma.

**Methods:**

80 asthma and 80 healthy controls were recruited in this study. The peripheral blood mononuclear cells (PBMCs) and serum samples of the asthma patients as well as the healthy controls were isolated, and the expression levels of miR-3934 in PBMCs were examined by RT-qPCR methods. Furthermore, the relationship between the level of miR-3934 in PBMCs and the disease severity has been analyzed, and the potential diagnostic value of miR-3934 was evaluated by the receiver operating characteristics (ROC) curve. Finally, the expression level of IL-6, IL-8, and IL-33 have been detected using the ELISA kits, and Pearson's correlation analysis was performed to investigate the relationship between the level of miR-3934 in PBMCs and the serum expression of those inflammatory cytokines in asthma patients.

**Results:**

miR-3934 was dramatically decreased in PBMCs of the asthma patients, and miR-3934 was markedly reduced in PBMCs of patients with severe asthma vs. mild asthma. Furthermore, ROC analysis showed that levels of miR-3934 in PBMCs can distinguish asthma patient, especially the severe asthma patients from the controls. Finally, the levels of miR-3934 in PBMCs were negatively correlated with the serum levels of IL-6, IL-8, and IL-33 in asthma patients, respectively.

**Conclusions:**

miR-3934 was downregulated in PBMCs of asthmatic patients and may function as a potential diagnosis biomarker.

## 1. Introduction

Asthma is a common chronic airway inflammatory disease. In recent years, its incidence has been on the rise all over the world [1–3]. Severe asthma has seriously affected human health and increased socioeconomic burden [4, 5] The receptor for advanced glycation end products (RAGE) is a multiligand receptor that belongs to the immunoglobulin superfamily. Accumulating evidence has indicated that RAGE is considered a key mediator of asthma pathogenesis [6]. RAGE is highly expressed in the lung tissues of patients with various respiratory diseases including asthma [7–9]. It is speculated that inhibiting RAGE expression may play a role in reducing airway inflammation in asthma.

microRNA (miRNA) is a group of small noncoding RNAs, 18-25 nucleotides in length. They act as gene inhibitors by negatively regulating the expression of their target genes. Previous studies have shown that miRNA may play an important role in the pathogenesis of different diseases, such as cancer, cardiovascular diseases, and autoimmune diseases [10–13]. It has also been found that some miRNAs are abnormally expressed in asthma [14–18]; however, few studies have focused on the expression of miRNAs in PBMC of asthma patients and their possible underlying mechanisms.

First, with bioinformatics analysis (TargetScan), we noticed that miR-3934 is complementary to the 3′ untranslated region (UTR) in RAGE. The miR-3934 was verified by luciferase assay to bind with the sequence “ACACCUGA” in RAGE. Moreover, it was observed that the overexpression of miR-3934 can suppress the expression level of RAGE. Therefore, we predicted that miR-3934 may be a potential negative regulatory sequence for RAGE. Considering that the RAGE expression was significantly high in PBMCs from asthma patients, this study is aimed at investigating the potential clinical value of detecting the expression level of miR-3934 in the PBMC of patients with asthma.

## 2. Material and Methods

### 2.1. Patients

The study recruited 80 patients with asthma who were diagnosed in the Second Affiliated Hospital of Harbin Medical University between January 2018 and September 2019. At the same time, 80 healthy volunteers without a history of lung disease, allergies, or respiratory infections were used as a control group. This study does not include candidates with autoimmune diseases, heart disease, AIDS, and other serious or systemic diseases. The severity of asthma is defined according to the Global Asthma Management and Prevention Strategy (updated in 2018) as follows: (1) mild: asthma that is well controlled with as-needed reliever medication alone or with low-intensity controller treatment such as low dose ICS; (2) moderate: asthma that is well controlled with low dose ICS/LABA or with high/moderate dose ICS; (3) severe: asthma that requires high-dose ICS/LABA to prevent it from becoming “uncontrolled” or asthma that remains “uncontrolled” despite this treatment [19]. The ethics documents were obtained from the Ethics Committee of the Second Affiliated Hospital of Harbin Medical University. The study obtained the informed consent of all candidates. In addition, the clinical data was collected for analysis, including demographic information and peripheral blood cell. The blood samples were collected while diagnosing asthma. After centrifugation, the serum samples were stored in a refrigerator at -80°C for further analysis.

### 2.2. Quantitative Real-Time RT-PCR

Because asthma is an immune disease, our group focused on the roles of immune cells in asthma. Therefore, we focused on the expression of miRNA in PBMCs. The level of miR-3934 in PBMCs was detected by qRT-PCR. Briefly, PBMCs were separated from blood samples as previously described [20]. The total RNAs were extracted from cells using TRIzol reagent (Invitrogen) and then reverse-transcribed into cDNAs using PrimeScript RT Master Mix (Takara, Dalian, China). Furthermore, the Hairpin-it™ miRNAs qPCR Quantitation Kit (Takara, Dalian, China) was used for RT-PCR reactions. ABI 7900 Biosystems (Applied Biosystems Life Technologies, Foster City, USA) was used for amplification by the following program: 95°C for 30 secs, 40 cycles of 95°C for 5 secs, and 60°C for 30 secs. U6 was employed for normalization, and primers were designed by Genescript (Nanjing, China). The level of miR-3934 in each sample was quantified by the 2^−*ΔΔ*Ct^ method.

### 2.3. Enzyme-Linked Immunosorbent Assay

The expression level of IL-6, IL-8, and IL-33 in serum samples of asthmatic patients, as well as healthy subjects, were detected by the enzyme-linked immunosorbent assay (ELISA) using commercially available kits (Nanjing Jiancheng Bio-Engineering Institute Co., Ltd., Nanjing, China). Procedures strictly followed the manufacturer's instructions.

### 2.4. Statistical Analysis

Continuous variables were presented as the median (interquartile range), and categorical variables were described as number and percentage (%). Differences between two normal distribution groups were compared by Student's *t*-test using the GraphPad Prism v7.0 software (GraphPad Software, CA, USA). Receiver operating characteristics (ROC) curve analysis was applied to predict the potential diagnostic value of miR-3934 for asthma. Pearson's correlation analysis was used for correlation studies. Significance was considered when the *p* value was less than 0.05.

## 3. Results

### 3.1. Downregulation of miR-3934 in PBMCs of Asthmatic Patients Compared with Healthy Controls

The expression levels of miR-3934 in PBMCs of asthmatic patients and that of healthy volunteers were compared by RT-PCR analysis. There were no significant differences between the asthma group and the control group in terms of age, gender, smoke history, allergy history, and white blood cell count (Table 1, *p* > 0.05). It has been observed that miR-3934 expression was dramatically decreased in PBMCs of asthmatic patients in comparison with that of healthy controls (Figure 1, *p* < 0.001). Furthermore, patients were divided into a mild (*n* = 52) and severe group (*n* = 28) based on the severity of the disease as previously described [19]. The association between miR-3934 levels in PBMCs of patients and severity of the disease has also been analyzed. We found that compared with patients with mild asthma, miR-3934 levels markedly decreased in PBMCs of patients with severe asthma (Figure 1(b), *p* < 0.01).

### 3.2. Potential Diagnostic Value for Detecting miR-3934 Levels in PBMCs of Asthmatic Patients

The potential diagnostic values of miR-3934 for asthma were evaluated by receiver-operating characteristic curves (ROC). As Figure 2(a) shows, the area under curve (AUC) value for miR-3934 levels in PBMCs to distinguish asthmatic patients from healthy subjects was 0.8041 (Figure 2(a), 95% confidence interval (CI), 0.7366–0.8715). Moreover, when asthmatic patients were divided into mild and severe groups, the AUC value of miR-3934 was 0.7666, to distinguish between mild asthmatic patients from healthy subjects (Figure 2(b), 95% CI, 0.6880–0.8452), and 0.8737 to distinguish between severe asthmatic patients and healthy subjects (Figure 2(c), 95% CI, 0.8074–0.9399). The above results indicated that miR-3934 may serve as a sensitive biomarker for the early diagnosis of asthma, particularly for those with severe asthma.

### 3.3. Proinflammatory Cytokines Were Increased in Serum of Asthmatic Patients

Proinflammatory factors in all subjects, including IL-6, IL-8, and IL-33, were evaluated by ELISA. The results showed that the levels of IL-6, IL-8, and IL-33 were markedly increased in serum of patients with asthma in comparison with that of healthy subjects (Figure 3, *p* < 0.01).

### 3.4. Correlation between miR-3934 Expression in PBMCs and Serum Levels of IL-6, IL-8, and IL-33 in Asthmatic Patients

We performed Pearson's correlation analysis to analyze the relationship between the miR-3934 expression in PBMCs and serum levels of some proinflammatory cytokines in asthmatic patients (Figure 4). We found that the miR-3934 expression levels in PBMCs negatively correlated with serum expression of IL-6 (*r* = −0.3726, *p* = 0.0007), IL-8 (*r* = −0.3656, *p* = 0.0009), and IL-33 (*r* = −0.2323, *p* = 0.0381) in asthmatic patients, respectively.

## 4. Discussion

In the current work, we investigated the potential clinical significance of miR-3934 in asthma. The main finding is that miR-3934 is significantly reduced in PBMC of asthmatic patients, and the level of miR-3934 in PBMC can distinguish asthmatic patients from healthy controls. And the level of miR-3934 is negatively correlated with the severity of the disease. Finally, the level of miR-3934 in PBMCs is negatively correlated with the expression of certain inflammatory cytokines in the serum of asthma patients.

The roles of miRNAs in asthma have been discussed in previous work, e.g., miR-221 and miR-485-3p were upregulated in asthma and may serve as potential biomarkers [21]; miR-192-5p has been reported to attenuate remodeling of the airway as well as autophagy in asthma [14]. miR-3934 is a recently identified miRNA, and its role in asthma has not been discussed. The results of the bioinformative analysis showed that there are many miRNAs that target 3′UTR of RAGE. Based on the unpublished results of our group, miR-3934 is the most significantly differently expressed miRNA between patients and healthy controls; more importantly, the direct targeting relationship between miR-3934 and RAGE was confirmed by due luciferase report assay. Therefore, miR-3934 was selected as a target in the present study.

Although it is more convenient to examine the expression of miRNAs in the serum or plasma samples, there are many studies focused on miRNA expression as biomarkers in PBMCs in different diseases, especially for immune diseases. Since asthma is an immune disease, in the current study, miRNA levels in PBMCs of 80 patients and healthy controls were compared. The results showed that miR-3934 was downregulated in asthma. This suggested that miR-3934 might be involved in asthma pathogenesis. Moreover, ROC analysis confirmed that miR-3934 levels in PBMCs can distinguish between disease intensity of asthmatic patients, especially between severe asthmatic patients and healthy controls. Overall, our study revealed that miR-3934 levels in PBMCs may function as potential diagnostic markers for asthma. Screening the expression of miR-3934 in PBMC may help identify asthma patients who are prone to severe diseases. Preventive targeted therapy for these patients is expected to reduce the frequency of acute attacks and reduce the economic burden.

It has been widely accepted that asthma is an inflammatory disease, and inflammation has been considered an important event during the occurrence and progress of asthma [22–25]. Several cytokines were found to be abnormally expressed in asthma serum and are associated with disease development [22, 25]. IL-6, IL-8, and IL-33 are known as proinflammatory cytokines. In accordance with previous reports, we found that they markedly increased in asthmatic patients in comparison with healthy controls [19, 26–28]. Moreover, a negative correlation was observed between miR-3934 expressions in PBMCs and inflammatory cytokine levels. Interestingly, none of these proinflammatory cytokines has been predicted as the target gene of miR-3934. Therefore, we speculate that some important inflammatory regulators may be direct targets of miR-3934, and downregulation of miR-3934 in PBMC may be related to the expression of these molecules and consequentially activate inflammatory signaling and lead to increased expression of proinflammatory cytokines. In other words, the upregulation of miR-3934 in PBMC may play a protective role in the occurrence of asthma.

In this research, we focused on the clinical implication of miR-3934 in asthma, and its hypothesized mechanism, mainly through serological analyses. Furthermore, the targets of miR-3934 in asthma should be identified by performing cell and animal studies.

In conclusion, miR-3934 was downregulated in PBMCs of asthmatic patients and may function as a potential diagnostic marker. Although the current work needs to be further confirmed by larger sample size, the results of this study have proposed potential clinical implications of miR-3934 in early diagnosis and management of asthma.

## Figures and Tables

**Figure 1:** Downregulation of miR-3934 in peripheral blood mononuclear cells (PBMCs) of asthmatic patients. (a) Comparison of expression levels of miR-3934 in PBMCs of asthmatic patients and healthy controls. (b) Comparison of expression levels of miR-3934 in PBMCs of severe asthmatic patients and mild asthmatic patients. ^∗∗∗^*p* < 0.001, ^∗^*p* < 0.05.

**Figure 2:** Potential diagnostic value of miR-3934 in peripheral blood mononuclear cells (PBMCs) for asthma. (a). Receiver operating characteristic (ROC) analysis for miR-3934 to distinguish between asthmatic patients and healthy controls. (b) ROC analysis for miR-3934 to distinguish between mild asthmatic patients and healthy controls. (c) ROC analysis for miR-3934 to distinguish between severe asthmatic patients and healthy controls.

**Figure 3:** Interleukin-6 (IL-6), IL-8, and IL-33 were overexpressed in the serum of asthmatic patients. ^∗∗^*p* < 0.01.

**Figure 4:** Correlation between miR-3934 expression and levels of interleukin-6 (IL-6), IL-8, and IL-33 in asthmatic patients.

**Table 1:** Clinical characteristics of the asthma patients and controls.

	Asthma patients (*n* = 80)	Controls (*n* = 80)	*p* value
Gender—*n* (%) (male/female)	49 (61.25%)/31 (38.75%)	45 (56.25%)/35 (43.75%)	0.5206
Age—median (IQR)	32 (20,48)	35 (23-49)	0.4126
Smoking history—*n* (%) (yes/no)	44 (55%)/36 (45%)	40 (50%)/40 (50%)	0.5266
Allergy history—*n* (%) (yes/no)	9 (18%)/71 (82%)	0 (0%)/80 (100%)	0.3766
WBC—median (IQR) (normal range 4.0 ~ 10.0 × 10^9^/L)	6.6 (3.9-8.2)	7.3 (4.6-9.5)	0.5546
Eosinophil—median (IQR) (normal range 0.05 ~ 0.45 × 10^9^/L)	0.85 (0.23-1.56)	0.37 (0.12-0.46)	<0.05

Note: WBC: white blood cell.

## Data Availability

The data used to support the findings of this study are available from the corresponding author upon request.
